The article "Effects of Different Anesthetics on Perioperative Organ Protection and Postoperative Cognitive Function in Patients Undergoing Cardiac Valve Replacement with Cardiopulmonary Bypass" was retracted in 2023. Reasons: signs of a paper mill; suspected computer-generated content; unreliable results or conclusions; concerns about the data.

# Effects of Different Anesthetics on Perioperative Organ Protection and Postoperative Cognitive Function in Patients Undergoing Cardiac Valve Replacement with Cardiopulmonary Bypass

**DOI:** 10.1155/2022/8994946

**Published:** 2022-05-29

**Authors:** Shenglan Mei, Yifan Jia, Jinjian Zhou, Ling Zhan, Jin Liu, Hao Ming, Huagang Liu

**Affiliations:** ^1^Department of Anesthesiology, People's Hospital of Wuhan University, Wuhuna, China; ^2^Department of Pain, People's Hospital of Wuhan University, Wuhuna, China; ^3^Department of Vascular Surgery, People's Hospital of Wuhan University, Wuhuna, China

## Abstract

In this paper, we have carried out an experimental study to investigate the effects of different anesthetics on perioperative organ protection and postoperative cognitive function in patients undergoing cardiac valve replacement with cardiopulmonary bypass. To realize this idea, a total of 90 patients with single valve replacement under general anesthesia and hypothermic cardiopulmonary bypass from January 2020 to October 2021 were enrolled. These patients were assigned into three groups, with 30 cases in each group by the digital table method. Group A was anesthetized with sufentanil combined with dexmedetomidine. Group B was anesthetized with sufentanil combined with etomidate. Group C was anesthetized with sufentanil combined with propofol. Perioperative organ protection and postoperative cognitive function of the three groups were compared. At *T*_0_ time point, there was no significant difference in blood WBC, blood *N*, and CRP among groups A, B, and C (*P* > 0.05); At *T*_4_ and *T*_5_ time points, the indexes of blood WBC, blood *N*, and CRP in groups A, B, and C were higher compared to the *T*_0_ time point. At *T*_4_ and *T*_5_ time points, the indexes of blood WBC, blood *N,* and CRP in group A were significantly lower compared to group B and group C. Before treatment, there was no significant difference in ALT and AST among groups A, B, and C (*P* > 0.05). After treatment, the indexes of ALT and AST in group A were significantly lower compared to group B and group C at *T*_4_ and *T*_5_ time points (*P* < 0.05). Before treatment, there was no significant difference in urea and creatinine among groups A, B, and C (*P* > 0.05). After treatment, the urea and creatinine indexes of group A were significantly lower compared to group B and group C at *T*_4_ and *T*_5_ time points (*P* < 0.05). Before treatment, there was no significant difference in CK-MB and CTnl among groups A, B, and C (*P* > 0.05); After treatment, the indexes of CK-MB and CTnl in group A were significantly lower compared to group B and group C at *T*_4_ and *T*_5_ time points (*P*  < 0.05). Before treatment, there was no significant difference in MOCA scores among groups A, B, and C (*P* > 0.05). After treatment, the MOCA scores of group A were significantly higher compared to group B and group C at *T*_5_ and *T*_6_ time points (*P*  < 0.05). Sufentanil combined with dexmedetomidine for heart valve replacement under cardiopulmonary bypass can reduce the dosage of anesthetics during the operation and have a certain perioperative protective effect on important organs such as the heart, lung, liver, and kidney, which may be related to reducing intraoperative hemodynamic fluctuations and inhibiting inflammatory stress response.

The article "Effects of Different Anesthetics on Perioperative Organ Protection and Postoperative Cognitive Function in Patients Undergoing Cardiac Valve Replacement with Cardiopulmonary Bypass" was retracted in 2023. Reasons: signs of a paper mill; suspected computer-generated content; unreliable results or conclusions; concerns about the data.

## 1. Introduction

Valvular heart disease is a series of diseases that is caused by changes in the structure or function of the heart valve and the failure of normal blood circulation [1]. Rheumatic heart disease is the main cause of rheumatic heart failure in China. It is a chronic valvular disease, common in women, especially 20–40, caused by rheumatic valvulitis [2]. Mitral valve disease is common. [2]. The clinical manifestations are valvular insufficiency, stenosis resulting in increased cardiac load, and cardiac insufficiency [3]. A common treatment method for this disease is heart valve replacement for both middle and advanced level rheumatic heart disease, mainly replacing the diseased valve with an artificial valve to improve clinical symptoms, and the operation is usually carried out under cardiopulmonary bypass [4]. Cardiopulmonary bypass is the use of a special artificial device to draw blood from the superior vena cava, inferior vena cava, and right atrium back to the heart and lung machine for oxygen and carbon dioxide discharge and then through the blood pump to continue blood circulation [5]. However, the anesthetic tolerance of patients with this disease is poor, and the internal environment of the body is exposed to foreign bodies such as oxygenators and ducts during cardiopulmonary bypass, which can cause monocyte/macrophage activation, resulting in massive production of inflammatory cytokines and waterfall release [6]. Coupled with ischemia-reperfusion during cardiopulmonary bypass, multiple organ functions can be directly or indirectly damaged. The inflammatory stress response and organ ischemia-reperfusion injury can lead to further aggravation of organ injury, bringing about a systemic diffuse multiorgan inflammatory stress response. It may even cause acute failure of vital organs such as the liver, kidney, and lungs [7]. The incidence of postoperative complications is very high, and the most common complications are heart and brain injury. Related studies have indicated that the selection and compatibility of anesthetic drugs are closely related to postoperative complications [8].

The article "Effects of Different Anesthetics on Perioperative Organ Protection and Postoperative Cognitive Function in Patients Undergoing Cardiac Valve Replacement with Cardiopulmonary Bypass" was retracted in 2023. Reasons: signs of a paper mill; suspected computer-generated content; unreliable results or conclusions; concerns about the data.

In this paper, we have performed numerous experiments to investigate the effects of different anesthetics on perioperative organ protection and postoperative cognitive function in patients undergoing cardiac valve replacement with cardiopulmonary bypass. Moreover, a detailed description is provided on how selected patients are divided into various groups, i.e., A, B, and C.

The rest of the manuscript is arranged according to the following agenda items.

In the section entitled “Patient and Methods,” a detailed note is provided on how many patients were selected and how these patients were divided into various groups. Moreover, selection and rejection criteria were described in detail.

## 2. Patients and Methods

### 2.1. General Information

A total of 90 patients undergoing single valve replacement under hypothermic cardiopulmonary bypass under general anesthesia in our hospital from January 2020 to October 2021 were enrolled. And, the patients were assigned into three groups, with 30 patients in each group (*n* = 30). Group A was anesthetized with sufentanil combined with dexmedetomidine, group B was anesthetized with sufentanil combined with etomidate, and group C was anesthetized with sufentanil combined with propofol. Among these patients, the age of group A was 40–76 years, that of group B was 41–77 years, and that of group C was 40–75 years. There was no significant difference in sex, age, and other general data (*P* > 0.05), which was comparable, as indicated in Table 1. All patients were aware of the study plan and signed the consent form, which was permitted by the ethics committee of our hospital.

### 2.2. Nanoplatoon Standard

#### 2.2.1. Inclusion Criteria

The inclusion criteria were as follows: (1) informed consent of patients; (2) ASA was classified as II or III; (3) NYHA was classified as II or III; (4) patients with rheumatic and degenerative valvular diseases undergoing elective single valve replacement were all patients with primary valve replacement and left ventricular ejection fraction (EF) ≥45%; (5) years of education >7 years; (6) there was no myocardial infarction in recent 3 months; and (7) there was no severe heart failure and malignant arrhythmia, no uncontrollable hyperglycemia, and no hypertension.

#### 2.2.2. Exclusion Criteria

The exclusion criteria were as follows: (1) more than 75 years old or less than 35 years old; (2) previous history of the central nervous system and mental illness and recent use of psychotropic drugs; (3) patients with severe liver, kidney, lung, and brain dysfunction before operation; (4) preoperative sinus bradycardia with any grade of atrioventricular block; and (5) there was a history of a severe allergy to anesthetic drugs (propofol, atracurium cis-benzenesulfonate, dexmedetomidine, and opioid analgesics) and substitute plasma.

The article "Effects of Different Anesthetics on Perioperative Organ Protection and Postoperative Cognitive Function in Patients Undergoing Cardiac Valve Replacement with Cardiopulmonary Bypass" was retracted in 2023. Reasons: signs of a paper mill; suspected computer-generated content; unreliable results or conclusions; concerns about the data.

### 2.3. Intervention Method

Group A was anesthetized with sufentanil combined with dexmedetomidine. Routine fasting before operation, ECG monitoring after entering the room, oxygen inhalation by mask, and establishment of venous access were carried out. Arterial blood pressure was monitored by radial artery catheterization. Right medetomidine, 0.4 *μ*g/(kg/h), was injected intravenously before induction and maintained until the end of operation. Then, anesthesia induction began. Midazolam, 0.02–0.05 mg/kg; etomidate, 0.2–0.3 mg/kg; and atracurium cis-sulfonate, 0.15–0.3 mg/kg, were injected intravenously, and sufentanil, 0.5–1 *μ*g /kg, was given. Mechanical ventilation was performed after intubation, and central venous pressure was monitored during the operation. After induction, midazolam, 0.05 mg/(kg/h); atracurium cis-benzenesulfonate, 0.1 mg/(kg/h); and sufentanil, 0.5–1 mg/(kg/h), were injected intravenously. During the operation, the drug concentration was adjusted according to the patient's blood pressure and heart rate. Group B was anesthetized with sufentanil combined with etomidate. Etomidate 0.2–0.4 mg/kg was injected intravenously before induction and maintained until the end of the operation. Group C was anesthetized with sufentanil combined with propofol—target-controlled infusion of propofol, the initial plasma target concentration of 1 *μ*g/ml, increased by 0.3 *μ*g/ml. Others are the same as group A.

### 2.4. Observation Index

#### 2.4.1. Index of Inflammatory Stress Response before and after Operation

Venous blood samples were taken 1 day before entering the operating room (T0), 1 day after the operation (T4), 3 days after the operation (T5), and 7 days after the operation (T6) to detect the expression of inflammatory factors such as WBC, *N*%, CRP, and hs-CRP.

#### 2.4.2. Organ Protection Index before and after Operation

Detection of clinical indicators commonly used to measure organ function mainly include liver function index ((alanine aminotransferase (ALT) and aspartate aminotransferase (AST)), renal function index (urea (UREA), creatinine (CREA), and cystatin C (CysC)), and cardiac function index (creatine kinase isoenzyme MB (CK-MB) and troponin I (cTnI)). The oxygenation index (OI) and alveolar-arterial oxygen partial pressure difference (*P* similar to aD02) were calculated for clinical evaluation of pulmonary function. The formula for calculating the alveolar-arterial oxygen partial pressure difference is *P* (A-aDO_2_) is *P* (A-aDO_2_) = (PB-PH20) × FiO_2_−PaCO_2_/R-PaO_2_, where PB is atmospheric pressure (760 mmHg) and PH20 is 37. At C, saturated water vapor pressure (47 mmHg), *R* is respiratory quotient (0.8), that is, alveolar-arterial oxygen partial pressure difference (A-aDO_2_) = 713 × FiO_2_−PaCO_2_ × 1.25−PaO_2_; oxygenation index: OI = PaO_2_/FiO_2_.

The article "Effects of Different Anesthetics on Perioperative Organ Protection and Postoperative Cognitive Function in Patients Undergoing Cardiac Valve Replacement with Cardiopulmonary Bypass" was retracted in 2023. Reasons: signs of a paper mill; suspected computer-generated content; unreliable results or conclusions; concerns about the data.

### 2.5. Statistical Methods

All data were analyzed by SPSS20.0 software. Among them, the measurement data are expressed as a *t*-test, the counting data are expressed by the number of cases (%), the *χ*^2^ test is used, and the grade data are expressed by a rank-sum test, expressed by *U*, and the difference exhibits significant (*P* < 0.05).

## 3. Results

### 3.1. Comparison of Inflammatory Stress Response Indexes before and after Operation

There was no significant difference in blood WBC, *N*, and CRP among groups A, B, and C at *T*_0_ time point, but at *T*_4_ and *T*_5_ time points, blood WBC, *N*, and CRP in groups A, B, and C were all higher compared to *T*_0_ time point. At *T*_4_ and *T*_5_, the levels of WBC, *N,* and CRP in group A were significantly lower compared to group B and group C. The specific results are shown in Figure 1.

### 3.2. Organ Protection Index before and after Operation

Before treatment, there was no significant difference in ALT and AST among groups A, B, and C (*P* > 0.05). After treatment, the indexes of ALT and AST in group A at *T*_4_ and *T*_5_ were significantly lower compared to groups B and C (*P* < 0.05). Before treatment, there was no significant difference in UREA and CREA among groups A, B, and C (*P* > 0.05). After treatment, the indexes of UREA and CREA in group A at *T*_4_ and *T*_5_ were significantly lower compared to groups B and C (*P* < 0.05). Before treatment, there was no significant difference in CK-MB and cTnl among groups A, B, and C (*P* > 0.05). After treatment, the indexes of CK-MB and cTnl in group A at *T*_4_ and *T*_5_ were significantly lower compared to group B and group C (*P* < 0.05). The specific results are shown in Tables 2–4.

### 3.3. Evaluation of Cognitive Function of Patients

Before administering the prescribed treatment, there was no significant difference in MoCA scores among groups A, B, and C (*P* > 0.05). After treatment, the MoCA scores of patients in group A at *T*_5_ and *T*_6_ were significantly higher compared to group B and group C (*P* < 0.05). The results are shown in Figure 2.

## 4. Discussion

With the increase of cardiovascular diseases in China, the cases of cardiac arrest and CPR are also increasing [9]. Although the CPR guidelines are constantly updated, the incidence of multiple organ dysfunction syndrome after resuscitation is very high due to ischemia-reperfusion injury, which seriously affects the prognosis [10]. Patients after CPR often experience multiple organ dysfunction due to increased oxygen consumption, disturbance of oxygen uptake and utilization, and apoptosis caused by inflammatory reactions and sympathetic excitement. Dexmetomidine can protect the function of important organs by inhibiting inflammatory reactions, antisympathetic activity, apoptosis, and other ways [11]. At present, dexmedetomidine and sufentanil are commonly adopted anesthetic drugs in clinics, and they are widely adopted, but the previous domestic studies on the combination of the two drugs are mainly focused on animal experimental studies, mainly on the clinical application of their combination in ICU patients, abdominal surgery, gynecological surgery, thoracic surgery, orthopedic surgery, etc., and mostly study their analgesic and sedative effects [12]. Research on the application of the combination of the two drugs in cardiovascular surgery is mainly focused on its effects on hemodynamics, analgesia, and sedation in elderly patients with coronary artery disease during coronary artery bypass surgery [13]. There are few reports on its protective effects on inflammatory stress response and organ injury induced by valve replacement under cardiopulmonary bypass [14, 15].

The article "Effects of Different Anesthetics on Perioperative Organ Protection and Postoperative Cognitive Function in Patients Undergoing Cardiac Valve Replacement with Cardiopulmonary Bypass" was retracted in 2023. Reasons: signs of a paper mill; suspected computer-generated content; unreliable results or conclusions; concerns about the data.

During cardiac valve replacement under cardiopulmonary bypass, direct exposure to the internal environment leads to inflammatory factors, monocyte (macrophage) activation, and immune rejection, resulting in multiple organ dysfunction [13]. Meanwhile, it may also be due to mechanical stimulation such as endotracheal intubation, arrhythmia, elevated blood pressure, and other hemodynamic symptoms. Stable body condition during the operation is helpful to reduce related complications [16]. Sufentanil is an opioid agonist derived from fentanyl, which has better lipophilicity than fentanyl and is easy to combine with plasma protein, so sufentanil can prolong the anesthetic time to ensure efficacy and help to maintain the stability of various indexes of the body. However, the intraoperative awareness rate of patients treated with drugs alone is likely to occur [17]. Dexmedetomidine is a new type of *α* 2-adrenergic receptor agonist and an imidazole derivative. It has extensive and stable sedation, analgesia, and antianxiety effects and has mild respiratory inhibition and little effect on hemodynamics. Some studies have indicated that sufentanil combined with dexmedetomidine can effectively enhance heart and brain injury, stabilize hemodynamics, coordinate analgesia and sedation, and reduce the dosage of anesthetics and analgesics in patients undergoing cardiac valve replacement under cardiopulmonary bypass [18]. Etomidate acted quickly had no significant effect on heart rate after anesthesia, slightly dilated coronary vessels to increase coronary blood flow, had no inhibitory effect on respiration, had no obvious drug toxicity, and reduced myocardial oxygen consumption [19]. Sufentanil and etomidate had inhibitory effects on cardiovascular and autonomic nervous function, but the inhibitory effect of etomidate was less than that of sufentanil, which combined with etomidate not only had a strong sedative effect but also had little effect on the circulatory system, but had a weak inhibitory effect on mechanical stimuli such as endotracheal intubation. The hemodynamic indexes changed significantly during intubation [20]. Propofol is a rapid and powerful anesthetic, which has the advantages of quick effect, no accumulation after continuous infusion, and quick recovery. Propofol is the first choice for clinical anesthesia and is widely adopted in surgical anesthesia and sedation therapy [21]. However, propofol can reduce sympathetic excitability, dilate blood vessels, and inhibit myocardial hypotension, so the anesthetic dose and infusion mode should be strictly controlled. During valve replacement under cardiopulmonary bypass, sufentanil combined with propofol is usually anesthetized by target-controlled infusion, which uses plasma blood on the basis of pharmacokinetics and pharmacodynamics. Anesthetic precautions for cardiac valve replacement: a comprehensive evaluation was given to patients before anesthesia, including medical history, relevant examination results, and disease severity, in order to predict patients' exposure to anesthesia and surgical risks, formulate anesthesia plans and countermeasures, and closely monitor patients' important physiological indexes during anesthesia. Mitral stenosis replacement should prevent tachycardia and decreased cardiac output, prevent bradycardia and hypotension, ensure sufficient blood volume to control infusion speed and dose, and avoid pulmonary edema. Digitalis should be given to control heart rate when atrial fibrillation or ventricular rate is too fast [22]. Mitral regurgitation replacement should prevent hypertension from increasing regurgitation, give dilators to reduce peripheral resistance, maintain sufficient blood volume, properly give positive inotropic drugs to support left ventricular function, and avoid increased pulmonary artery pressure caused by hypoxia, carbon dioxide accumulation, and acidosis. During aortic valve stenosis replacement, sinus rhythm should be maintained, proper intravascular volume should be maintained, hypotension should be prevented, and vasoconstrictor should be given appropriately when blood pressure drops, and drugs should be given before anesthesia to reduce tachycardia and agitation to avoid myocardial ischemia; intraoperative infusion maintains left ventricular filling pressure; pacemakers were placed in patients with loss of sinus rhythm or atrial degeneration [23]. Aortic valve insufficiency replacement should prevent increased peripheral resistance, bradycardia, and other aggravating factors of regurgitation; appropriate administration of vasodilators to increase forward blood flow; reduce peripheral resistance to reduce regurgitation; and maintain sufficient blood volume. The ideal clinical anesthetic state should achieve the purpose of quick effect, short effect, and mild inhibition in cardiovascular and respiratory function, which cannot be met by an anesthetic alone. At present, sufentanil is mainly used in valve replacement under cardiopulmonary bypass combined with other anesthetic drugs. In clinical practice, the selection and compatibility of anesthetics should make a reasonable anesthetic scheme according to the possible adverse reactions of combined administration and the condition of the patients, so as to achieve the best anesthetic effect and reduce body injury.

The article "Effects of Different Anesthetics on Perioperative Organ Protection and Postoperative Cognitive Function in Patients Undergoing Cardiac Valve Replacement with Cardiopulmonary Bypass" was retracted in 2023. Reasons: signs of a paper mill; suspected computer-generated content; unreliable results or conclusions; concerns about the data.

## 5. Conclusion

In this paper, we have carried out an experimental study to investigate the effects of different anesthetics on perioperative organ protection and postoperative cognitive function in patients undergoing cardiac valve replacement with cardiopulmonary bypass. Sufentanil combined with dexmedetomidine can reduce the amount of anesthetic during cardiac valve replacement under cardiopulmonary bypass and has a certain perioperative protective effect on the heart, lung, liver, kidney, and other important organs of the body. This may be related to the reduction of intraoperative hemodynamic fluctuations and the inhibition of inflammatory stress response, and it is safe. Limited by the sample size, the results of this study need to be confirmed by the enlarged central test.

## Figures and Tables

**Figure 1:** Comparison of inflammatory stress response indexes.

**Figure 2:** Assessment of cognitive function of patients.

**Table 1:** The comparison of general data between two groups.

Group	*N*	Gender (male/female)	Age (years)	NYHA grading	
				II	III
Group A	30	14/16	61.23 ± 7.23	18	12
Group B	30	15/15	60.75 ± 6.72	17	13
Group C	30	14/15	61.53 ± 7.14	17	13

**Table 2:** Comparison of protective indexes of liver injury before and after operation (${}^{\bar{x}\pm s}$, d).

	Group	*N*	*T*_0_	*T*_4_	*T*_5_
ALT (U/L)	Group A	30	36.32 ± 8.43	70.33 ± 7.26	61.42 ± 6.26
	Group B	30	36.26 ± 8.52	80.53 ± 10.45	74.53 ± 8.35
	Group C	30	37.16 ± 8.63	78.43 ± 8.92	71.24 ± 5.36

AST (U/L)	Group A	30	29.41 ± 7.32	62.42 ± 9.24	54.53 ± 7.37
	Group B	30	29.53 ± 7.14	71.35 ± 10.25	65.38 ± 8.58
	Group C	30	29.46 ± 7.37	67.53 ± 10.17	61.38 ± 9.15

The article "Effects of Different Anesthetics on Perioperative Organ Protection and Postoperative Cognitive Function in Patients Undergoing Cardiac Valve Replacement with Cardiopulmonary Bypass" was retracted in 2023. Reasons: signs of a paper mill; suspected computer-generated content; unreliable results or conclusions; concerns about the data.

**Table 3:** Comparison of observation indexes of renal injury protection before and after operation (${}^{\bar{x}\pm s}$, d).

	Group	*N*	*T*_0_	*T*_4_	*T*_5_
UREA (mmol/L)	Group A	30	5.56 ± 1.02	9.02 ± 0.95	7.83 ± 0.61
	Group B	30	5.57 ± 1.12	11.79 ± 1.62	11.24 ± 1.52
	Group C	30	5.70 ± 1.32	11.21 ± 1.72	10.46 ± 1.57

CREA (*µ*mol/L)	Group A	30	90.53 ± 6.92	246.42 ± 62.42	200.41 ± 46.36
	Group B	30	90.42 ± 6.37	314.24 ± 68.42	267.43 ± 67.43
	Group C	30	91.02 ± 6.58	302.52 ± 66.73	254.64 ± 63.26

**Table 4:** Comparison of observation indexes of cardiac injury protection before and after operation (${}^{\bar{x}\pm s}$, d).

	Group	*N*	*T*_0_	*T*_4_	*T*_5_
CK-MB (ng/ml)	Group A	30	2.64 ± 0.89	43.53 ± 2.89	26.74 ± 3.46
	Group B	30	2.74 ± 1.02	48.10 ± 4.53	39.73 ± 4.25
	Group C	30	2.56 ± 0.98	47.83 ± 4.25	38.24 ± 3.84

cTnl (ng/ml)	Group A	30	0.28 ± 0.05	1.42 ± 0.07	1.01 ± 0.04
	Group B	30	0.29 ± 0.05	1.84 ± 0.08	1.48 ± 0.06
	Group C	30	0.28 ± 0.05	1.78 ± 0.08	1.40 ± 0.05

## Data Availability

The datasets used and analyzed during the current study are available from the corresponding author upon reasonable request.
